The article "The added value of color parameter imaging for the evaluation of focal liver lesions with “homogenous hyperenhancement and no wash out” on contrast enhanced ultrasound" was published in 2024. Journal: Front Oncol.

# The added value of color parameter imaging for the evaluation of focal liver lesions with “homogenous hyperenhancement and no wash out” on contrast enhanced ultrasound

**DOI:** 10.3389/fonc.2023.1207902

**Published:** 2024-01-11

**Authors:** Zi-Nan Liang, Song Wang, Wei Yang, Hong Wang, Kun Zhao, Xiu-Mei Bai, Zhong-Yi Zhang, Wei Wu, Kun Yan

**Affiliations:** Department of Ultrasound, Key Laboratory of Carcinogenesis and Translational Research (Ministry of Education/Beijing), Peking University Cancer Hospital, Beijing, China

**Keywords:** contrast-enhanced ultrasound, color parameter imaging, focal liver lesion, prediction model, nomogram

## Abstract

**Objective:**

The purpose of this study was to investigate the added value of color parameter imaging (CPI) in the differential diagnosis of focal liver lesions (FLLs) with “homogeneous hyperenhancement but not wash out” on contrast-enhanced ultrasound (CEUS).

**Methods:**

A total of 101 patients with 108 FLLs were enrolled in this study. All the FLLs received US and CEUS examinations. The stored CEUS clips of target lesions were postprocessed with CPI analysis by radiologists. The receiver operator characteristic (ROC) curve was used to evaluate the added value of CPI. The McNamara test was used to compare the diagnostic sensitivity, specificity, and accuracy between CEUS and CPI patterns. Univariate and multivariate logistic regression analyses were used to develop a CPI nomogram. The C index and calibration curve were used to evaluate the predictive ability of the nomogram. The intraclass correlation coefficient was used to test the reproducibility and reliability of CPI. Decision curve analysis (DCA) was used to evaluate the added value of applying CPI.

**Results:**

The following CPI features were more frequently observed in malignant FLLs: eccentric perfusion (malignant: 70.0% vs. benign: 29.2%, *p* < 0.001), feeding artery (51.7% vs. 4.2%, *p* < 0.001), mosaic (63.3% vs. 6.3%, *p* < 0.001), red ingredients >1/3 (90.0% vs. 14.6%, *p* < 0.001). In addition, centripetal (43.8% vs. 18.3%, *p* = 0.004), peripheral nodular (54.2% vs. 1.7%, *p* < 0.001), subcapsular vessel (12.5% vs. 0.0%, *p* = 0.004), spoke-wheel vessels (25.0% vs. 5.0%, *p* = 0.003), branched vessels (22.9% vs. 5.0%, *p* = 0.006), blue and pink ingredients >2/3 (85.4% vs. 10.0%, *p* < 0.001) were more observed in benign FLLs. A nomogram incorporating peripheral nodular, spoke-wheel vessels, and red ingredients >1/3 was constructed. The model had satisfactory discrimination (AUC = 0.937), and the optimal diagnostic threshold value was 0.740 (0.983, 0.850). By the DCA, the model offered a net benefit over the treat-all-patients scheme or the treat-none scheme at a threshold probability 5%–93%.

The article "The added value of color parameter imaging for the evaluation of focal liver lesions with “homogenous hyperenhancement and no wash out” on contrast enhanced ultrasound" was published in 2024. Journal: Front Oncol.

**Conclusion:**

Using CPI can detect and render subtle information of the main features of FLLs on CEUS; it is conducive to the radiologist for imaging interpretation, and a combining read of the CEUS and CPI of the FLLs with features of “homogenous hyperenhancement and no washout” can improve significantly the diagnostic performance of CEUS for FLLs.

## Introduction

Contrast-enhanced ultrasound (CEUS) can provide a real-time, dynamic enhancement pattern for focal liver lesions (FLLs) and provide information about lesion perfusion and vascularity. Therefore, CEUS significantly improves the differential diagnosis in FLLs (1, 2). The typical enhancement patterns for malignant FLLs (M-FLLs) are washed in at the arterial phase and washed out in the portal venous or late phase (3). For example, hepatocellular carcinoma (HCC) has this enhancement pattern on CEUS (4). According to previous research, 27.6% HCC exhibited no washout in the late phase (5), which is similar to some benign FLLs (B-FLLs). Some B-FLLs have some unique arterial phase features, such as hepatic hemangioma with peripheral nodular enhancement and focal nodular hyperplasia (FNH) with spoke-wheel enhancement (4). Due to the small size of the FLL or the perfusion features, some B-FLLs enhanced rapidly within a few seconds in the arterial phase, which is similar to that of M-FLL. It is very challenging to distinguish tiny differences in vascular hemodynamics by visual observation on CEUS in such a short time. It is difficult to distinguish between malignant and B-FLL with “homogenous hyperenhancement and no wash out” by CEUS alone.

Color parameter imaging (CPI) is customized software developed for the post-process of CEUS and improving characterization. It has been built-in exclusively into the US systems manufactured by the GE Healthcare (Chicago, IL, USA). It displays the arrival time of contrast agent microbubbles in the liver and lesions by arbitrary colors. CPI has the advantages of exhibiting more sufficiently the enhancement characteristics of CEUS for tissues and organs such as blood perfusion, direction and distribution of lesions and surrounding liver tissue in a detailed, and visualizable and real-time manner. CPI provides more hemodynamic features, which compensates for the shortcoming of visual observation in the arterial phase. Recently, several studies have reported CPI in the examination of FLLs and lymph nodes (6–12). According to previous studies, CPI could differentiate hepatic adenoma and FNH from HCC and can differentiate atypical hepatic hemangioma from liver metastases (6, 7, 11). CPI could predict the pathological classification of HCC and evaluate the radiofrequency ablation outcome of the tumor (10). To our knowledge, this is the first study focusing on the use of CPI technique in the differential diagnosis of FLLs with “homogeneous hyperenhancement in the arterial phase and no washout in the late phase.”

The article "The added value of color parameter imaging for the evaluation of focal liver lesions with “homogenous hyperenhancement and no wash out” on contrast enhanced ultrasound" was published in 2024. Journal: Front Oncol.

The aim of this study was to evaluate the role of CPI in the differential diagnosis of FLLs with “homogeneous hyperenhancement and no washout in the late phase” on CEUS.

## Materials and methods

### Patients

This retrospective study was approved by the institutional review board of the Peking University School of Oncology (2021KT77). Written informed consent for CEUS examination was obtained for all patients. Data collection and analysis received institutional review board approval, and the requirement for informed consent was waived.

From January 2018 to July 2021, a total of 2,913 patients with FLLs underwent CEUS examination in our department. The inclusion criteria were as follows: (a) patients aged between 18 years and 80 years, (b) the target lesions had no previous treatment, (c) the target lesions displayed homogenous hyperenhancement during the arterial phase and were not washed out during the late phase in CEUS, (d) the examination of the target lesions was performed by a Logiq E9 ultrasonic system, and (e) the target lesions had a final diagnosis. M-FLLs with the final diagnosis were confirmed by pathology (*n* = 31) and clinical diagnosis according to guidelines (*n* = 29) (13). B-FLLs were confirmed by pathology (*n* = 35) and contrast-enhanced computed tomography or magnetic resonance imaging results with at least 1 year of follow-up (*n* = 13). The exclusion criteria were as follows: (a) the target lesions were invisible during the examination and (b) low-quality imaging due to deep breath movement during the examination. Finally, 101 patients with 108 FLLs were enrolled in this study, including 60 M-FLLs and 48 B-FLLs (**Figure 1**). All of the M-FLLs were HCCs. Twenty-five of 31 pathologically confirmed lesions were well-moderately differentiated HCCs, and six of 31 lesions were poorly differentiated HCCs. The 48 B-FLLs included 27 hepatic hemangiomas, 14 FNHs, and seven hepatic adenomas.

**Figure 1:** Flow diagram of the study population. FLL , focal liver lesion; CEUS , contrast-enhanced ultrasound; AP , arterial phase; PVP , portal venous phase; LP , late phase; US , ultrasound; CPI , color parameter imaging; HCC , hepatocellular carcinoma; FNH , focal nodular hyperplasia.

### CEUS examination methods

Conventional US and CEUS examinations were performed by a Logiq E9 ultrasonic system (GE Healthcare, Chicago, IL, USA) with a C1-5 wide-band convex probe (2–5 MHz). The US contrast agent was SonoVue^®^ (sulphur hexafluoride microbubbles for injection) (Bracco Suisse SA, Switzerland; Shanghai Bracco Sine Pharmaceutical Corp. Ltd, China). The microbubbles suspension was prepared before use by injecting 5 mL of sodium chloride 0.9% solution to the contents of the vial. The vial is then shaken slightly for a few seconds to enable the contents in the vial dispersed completely, and a homogeneous white milky suspension was obtained. Before CEUS, the patient was trained to control breath to reduce the changes caused by breath activity. The specific operation process was as follows: (1) the location of the FLL was found and fixed at the best display section. (2) The US contrast mode was switched, and the dual-amplitude contrast mode was activated. The patient was instructed to keep still and control his or her breath (no deep breath) during the arterial phase. The mechanical index was set at 0.11–0.13. (3) A 1.5-mL dose of contrast agent was bolus injected into the antecubital vein via a 20-G cannula within 2–3 s, followed by a 5-mL saline flush. After the injection, the contrast harmonic imaging was performed with a timer initiated simultaneously. Dynamic intralesional blood perfusion was observed continuously from the arterial phase to the late phase of perfusion. Consecutive video clips (the 90 s for each clip) were recorded and stored on the hard disk for further analysis. Several video clips of every lesion were stored until 360 s after contrast agent injection. The arterial phase started at 10–20 s and ended at 30–45 s, the portal venous phase started at 30–45 s and ended at 120 s, and the late phase started at 120 s and ended at 4–8 min (4). These CEUS examinations were performed by experienced radiologists (Yang W, Wu W, and Zhang ZY with more than 5 years of CEUS experience).

The article "The added value of color parameter imaging for the evaluation of focal liver lesions with “homogenous hyperenhancement and no wash out” on contrast enhanced ultrasound" was published in 2024. Journal: Front Oncol.

### Color parameter imaging analysis

The stored CEUS clips of target lesions were tailored from the time of contrast agent injection to the peak time before CPI analysis. One radiologist (Wang H) color coded the tailored video using the CPI software onboard the Logiq E9 XD Clear US system (GE Healthcare, Chicago, IL, USA). In the CPI images, the color map consisted of individual pixels, representing the arrival time of the contrast agent. The injection time of the contrast agent was set as zero. The color and duration time could be adjusted. We established a color model representing vascular hemodynamics of FLLs based on the utility instruction manual for CPI software and our previous study (10). This color model of the CPI system consisted of four colors (red, blue, pink, and purple) according to the enhancing time sequence: (1) red [the contrast agent arrival time to hepatic artery (HA) to the arrival time of portal vein (PV) for the evaluation of the arterial phase enhancement], (2) blue [from the arrival time of PV to the time when the tumor was filled (greater than 90%) for the evaluation of the PV phase enhancement], (3) pink (2 s after blue that enabled depiction of the tumor margin), and (4) purple (started at the arrival time of adjacent liver parenchyma). The time axis was set individually to reduce individual differences in perfusion time. The setting of this time axis is basically consistent with other related literature (10). At the beginning of this study, we randomly selected 10 cases of tailored clips of video, processed using CPI and analyzed the CPI features of these FLLs in three times, and calculated intraclass correlation coefficients (ICCs).

### Evaluation of CEUS and CPI

The CEUS and CPI videos were read retrospectively and independently by two senior radiologists (Yang W and Wu W) with at least 15 years of experience in the evaluation of liver CEUS and by two junior radiologists (Liang ZN and Wang S) with more than 1 year of experience in liver CEUS. The two radiologists in the senior group reviewed the images and videos together and made consensus statements, so did the two radiologists in the junior group. When diagnosing FLL by CPI +CEUS imaging or CEUS, all the radiologists were blinded to the patient pathologic results and other imaging results.

According to the previous reports and our analysis, the characteristics of CPI were summarized as follows: (a) centripetal perfusion: enhanced from the periphery to the center; (b) eccentric perfusion: enhanced from one side to another side; (c) centrifugal perfusion: enhancement started from the center to the periphery; (d) peripheral nodular enhancement: round or semicircle-shaped enhancement visualized at the peripheral area of lesions; (e) feeding artery: hypertrophic vessel directed toward the tumor that was substantially larger than other vascular branches at the same depth (2 mm–3 mm in diameter); (f) subcapsular vessel: thick and tortuous blood vessel under the tumor capsule; (g) spoke-wheel vessels: arteries with a spoke-wheel or starlike morphology in the center of the lesion during the arterial phase; (h) mosaic enhancement: one or more hypertrophic tortuous arteries that reached the edge of the lesion, partially encircling the nodule and penetrating internally with a basket or chaotic distribution; (i) branched vessels: hypertrophic tortuous vessels with a few branches or dendritic vessels; and (j) blue and pink ingredients>2/3 or red ingredients >1/3 (**Figure 2**) (6, 7, 10, 11, 14).

The article "The added value of color parameter imaging for the evaluation of focal liver lesions with “homogenous hyperenhancement and no wash out” on contrast enhanced ultrasound" was published in 2024. Journal: Front Oncol.

**Figure 2:** Figures from the rows up to down illustrate or show the perfusion characteristics of different focal liver lesions with “homogenous hyperenhancement and no wash out” on diagrams, images of color parameter imaging, and images of contrast-enhanced ultrasound. The figures in the first row are diagrams of the perfusion characteristics of different focal liver lesions with “homogenous hyperenhancement and no wash out.” The figures in the second row are color parameter imaging corresponding to the patterns. The figures in the third row are routine contrast-enhanced ultrasound images. A1–A3, hepatic hemangioma; BI–B3, hepatocellular carcinoma; C1–C3, hepatocellular carcinoma; D1–D3, hepatic hemangioma; E1–E3, hepatocellular carcinoma; F1–F3, hepatic adenoma; G1–G3, focal nodular hyperplasia.

Both senior and junior radiologists were required to score the diagnosis of CEUS or CPI+CEUS, which used a 5-point scale: 1 = *benign with strong probability*, 2 = *probable benign*, 3 = *undetermined*, 4 = *probable liver malignancy*, and 5= *liver malignancy with strong probability* (11).

### Statistical analysis

SPSS Statistics for Windows, Version 24.0. (Armonk, NY: IBM Corp, USA), MedCalc software (MedCalc 19.2.1; MedCalc, Mariakerke, Belgium) and R version 4.1.2 (R Foundation for Statistical Computing, Vienna, Austria) were used for statistical analysis. Count data were analyzed by using the χ2 test and Fisher’s exact test. Tumor size was analyzed by the Mann−Whitney U test. The Kappa test was used to analyze the interrater agreement between the senior and junior radiologists. The agreement was graded as follows: moderate (0.2–0.39), fair (0.40–0.59), good (0.60–0.79), and perfect (0.80–1.0) agreement (11). The ICC was used to test the reproducibility and reliability of CPI.

According to the results of the univariate analysis of the senior group, multivariate logistic analysis was performed to identify independent predictors. Backward stepwise selection was applied to select the independent predictors for constructing the prediction model. A nomogram was established for differentiating benign and M-FLLs. The bootstrap was used to iterate 100 times for internal validation. The C index and calibration curve were used to evaluate the predictive ability of the nomogram. Decision curve analysis (DCA) was used to evaluate the added clinical application value of CPI.

Receiver operating characteristic curves and under the receiver operating characteristic curve (AUC) were plotted to evaluate the diagnostic performance of the discrimination between malignant and B-FLLs. Differences in AUCs were assessed by using the method described by Hanley and McNeil. The McNamara test was used to compare the diagnostic sensitivity, specificity, and accuracy between CEUS and CPI patterns. A *P*-value less than 0.05 was considered statistically significant.

The article "The added value of color parameter imaging for the evaluation of focal liver lesions with “homogenous hyperenhancement and no wash out” on contrast enhanced ultrasound" was published in 2024. Journal: Front Oncol.

## Results

### Clinical characteristics

A total of 101 patients with 108 FLLs were enrolled in this study, including 60 M-FLLs and 48 B-FLLs. The clinical characteristics of 108 FLLs were summarized in **Table 1**. The median diameters of the malignant and B-FLLs were 1.9 cm (range: 0.9 cm–6.4 cm) and 2.0 cm (range: 1.1 cm–10.2 cm) (*p* = 0.75), respectively. No significant difference was found in the clinical features between the malignant and B-FLLs, except for HBV/HCV infection (*P* < 0.001).

**Table 1:** The clinical characteristics of patients with malignant or benign focal liver lesions.

	M-FLL	B-FLL	*P*-value
Number of lesions	60	48	
Number of patients	55	46	
Sex			
Male	37	26	0.267
Female	18	20	
Age (year)	61.8 ± 10.6	47.9 ± 13.4	0.10
Tumor size (cm)	1.9	2.0	0.747
HBV/HCV	46	11	< 0.001
AFP			
> 200 μg/mL	7	4	0.517
< 200 μg/mL	48	42	
ALT/AST			
> 50 μg/mL	10	6	0.481
< 50 μg/mL	45	40	

M-FLL, malignant focal liver lesion; B-FLL, benign focal liver lesion.

### Consistency of CPI features and FLLs

The interobserver agreement for both the senior and junior groups for CPI were listed in **Table 2**. The interobserver agreement for the CPI features was mostly good and perfect, with *k*-values ranging from 0.724 ± 0.069 to 0.904 ± 0.095. The ICCs for CPI findings of FLLs listed in **Table 3**. In 70% lesions, the features obtained and observed at 3 times were completely consistent; all the values of ICC were 1. In 30% lesions, the values of ICC were excellent, with ranging from 0.830 to 0.877.

**Table 2:** Interobserver agreement of CPI features between senior and junior radiologists.

Feature	Kappa value
Centripetal	0.747 ± 0.068
Eccentric	0.778 ± 0.060
Centrifugal	0.746 ± 0.085
Peripheral nodular	0.848 ± 0.060
Feeding artery	0.749 ± 0.071
Subcapsular vessel	0.904 ± 0.095
Mosaic/chaotic	0.724 ± 0.069
Spoke-wheel vessels	0.789 ± 0.091
Branched vessels	0.813 ± 0.090
Blue and pink ingredients > 2/3 Red ingredients > 1/3	0.777 ± 0.061

CPI, color parameter imaging.

**Table 3:** The intraclass correlation coefficient for CPI findings of FLLs.

FLL	ICC
**Lesion 1**	**1**
**Lesion 2**	**1**
**Lesion 3**	**0.877 (0.969, 0.964)**
**Lesion 4**	**1**
**Lesion 5**	**1**
**Lesion 6**	**0.845 (0.63, 0.954)**
**Lesion 7**	**0.830 (0.592, 0.950)**
**Lesion 8**	**1**
**Lesion 9**	**1**
**Lesion 10**	**0.877 (0.696, 0.964)**

CPI, color parameter imaging; FLL, focal liver lesion; ICC, intraclass correlation coefficient.

### Diagnostic performance of CEUS and CEUS+CPI for FLLs

The diagnostic sensitivity, specificity, accuracy, AUC values and Youden’s index of CEUS, and CEUS+CPI between benign and M-FLLs were calculated in **Table 4**. The receiver operator characteristic (ROC) curves of CEUS and CEUS+CPI were displayed in **Figure 3**. In both groups of radiologists, the AUCs of CEUS+CPI were significantly higher than those of CEUS alone (senior: 0.925 vs. 0.823, *p* = 0.037; junior: 0.818 vs. 0.653, *p* = 0.001). For junior radiologists, the specificity and accuracy of CEUS+CPI were improved compared with those of CEUS (0.780 vs. 0.659, *p* = 0.006; 0.815 vs. 0.676, *p* = 0.007). Additionally, the diagnostic performance of CEUS+CPI for junior radiologists was similar to that of CEUS for senior radiologists, and the AUC was very close (0.823 vs. 0.818, *p* = 0.520).

The article "The added value of color parameter imaging for the evaluation of focal liver lesions with “homogenous hyperenhancement and no wash out” on contrast enhanced ultrasound" was published in 2024. Journal: Front Oncol.

**Table 4:** Comparisons of diagnostic performances of CEUS and CEUS+CPI for focal liver lesions.

Criteria	Sensitivity	*P*-value	Specificity	*P*-value	Accuracy	*P*-value	AUC	*P*-value	Youden’s index
Benign and malignant									
S-CEUS	0.867	0.228^a^	0.812	0.289^a^	0.843	0.066^a^	0.823	**0.037^a^**	0.679
S-CEUS+CPI	0.919	0.505^b^	0.935	1.0^b^	0.926	0.628^b^	0.925	0.520^b^	0.846
J-CEUS	0.687	0.546^a^	0.659	**0.006^a^**	0.676	**0.007^a^**	0.653	**0.001^a^**	0.329
J-CEUS+CPI	0.845		0.780		0.815		0.818		0.629
Hepatic hemangioma									
S-CEUS	0.778	0.289	0.938	0.375	0.898	0.092	0.858	0.08	0.716
S-CEUS+CPI	0.926		0.975		0.963		0.951		0.901
J-CEUS	0.519	0.070	0.926	0.219	0.824	**0.013**	0.722	**0.008**	0.444
J-CEUS+CPI	0.741		0.975		0.917		0.858		0.716
FNH									
S-CEUS	0.500	0.125	0.969	0.250	0.909	**0.021**	0.734	0.097	0.469
S-CEUS+CPI	0.857		1.000		0.981		0.929		0.857
J-CEUS	0.429	0.219	0.948	1.000	0.882	0.581	0.688	**0.022**	0.376
J-CEUS+CPI	0.714		0.938		0.909		0.826		0.652
Hepatic adenoma									
S-CEUS	0.333	0.250	0.962	0.500	0.927	1.000	0.647	**0.021**	0.295
S-CEUS+CPI	0.833		0.981		0.972		0.907		0.814
J-CEUS	0.333	0.500	0.933	0.508	0.900	0.227	0.633	0.088	0.266
J-CEUS+CPI	0.667		0.962		0.945		0.814		0.628

CEUS, contrast-enhanced ultrasound; CPI, color parameter imaging; P-value is comparison of CEUS+CPI and CEUS. “^a^Comparison” refers to the comparison between CEUS+CPI and CEUS. “ ^b^Comparison” refers to the comparison between CEUS+CPI in junior radiologists and CEUS in senior radiologists. “S-” refers to senior; “J-” refers to junior. The bold values are statistically signi-ficant values that are less than 0.05.

**Figure 3:** ROC curves of CEUS and CEUS+CPI for the evaluation of malignant and benign FLLs, hepatic hemangioma, FNH, and hepatic adenoma by senior and junior radiologist, respectively. CPI, color parameter imaging; FLL, focal liver lesion, FNH, focal nodular hyperplasia. **(A)** The area under the receiver operating characteristic (ROC) curve (AUC) was calculated to assess the ability of CPI+CEUS and CEUS alone, to distinguish between malignant and benign focal liver lesions. The AUC values obtained for CEUS+CPI were 0.925 and 0.818, as determined by senior and junior radiologists, respectively. Similarly, the AUC values for CEUS alone were 0.823 and 0.653, as determined by senior and junior radiologists, respectively. **(B)** In the assessment of hepatic hemangioma, the AUC values for the CPI+CEUS by senior and junior radiologists were found to be 0.951 and 0.858, respectively. The AUC values for CEUS alone in diagnosing hepatic hemangioma by senior and junior radiologists were 0.858 and 0.722, respectively. **(C)** In the assessment of FNH, the AUC values for the CPI+CEUS by senior and junior radiologists were found to be 0.929 and 0.826, respectively. The AUC values for the CPI+CEUS by senior and junior radiologists were found to be 0.734 and 0.688, respectively. **(D)** In the assessment of hepatic adenoma, the AUC values for the CPI+CEUS by senior and junior radiologists were found to be 0.907 and 0.814, respectively. The AUC values for the CPI+CEUS by senior and junior radiologists were found to be 0.647 and 0.633, respectively.

The article "The added value of color parameter imaging for the evaluation of focal liver lesions with “homogenous hyperenhancement and no wash out” on contrast enhanced ultrasound" was published in 2024. Journal: Front Oncol.

### Diagnostic performance of CEUS and CEUS+CPI for benign FLLs

The value of CEUS+CPI for the differential diagnosis of B-FLLs such as hepatic hemangioma, FNH, and hepatic adenoma was improved compared with CEUS alone (**Table 4** and **Figure 3**). For hepatic hemangioma, the AUC and accuracy of CEUS+CPI were significantly higher than those of CEUS in the junior group (0.858 vs. 0.722, *p* = 0.008; 0.917 vs. 0.824, *p* = 0.013). For FNH, the AUC of CEUS+CPI was significantly higher than that of CEUS in the junior group (0.826 vs. 0.688, *p* = 0.022). Furthermore, the accuracy of CEUS+CPI was significantly higher than that of CEUS in the senior group (0.981 vs. 0.909, *p* = 0.021). For hepatic adenoma, the AUC of CEUS+CPI was significantly higher than that of CEUS in the senior group (0.907 vs. 0.647, *p* = 0.021). The AUC of CEUS+CPI in the junior group was higher than that of CEUS but only as a trend observed (0.814 vs. 0.633, *p* = 0.088).

### Diagnostic confidence by CEUS and CEUS+CPI

The distribution of the diagnostic confidence scores of CEUS and CEUS+CPI in senior and junior radiologists was displayed in **Figure 4**. The scores of CEUS+CPI imaging were mostly distributed on the definite diagnosis sites 1-score and 5-score of the senior radiologists (72.7%). The number of 1-scores and 5-scores between CEUS and CEUS+CPI was significantly different (senior: 28.8% vs. 4.6%, *p* < 0.001; 43.5% vs. 14.8%, *p* < 0.001; junior: 22.2% vs. 1.9%; 28.7% vs. 2.8%, *p* < 0.001 of all). In both groups of radiologists, the number of undetermined diagnoses (3-score) in CEUS+CPI was obviously lower than that in CEUS (senior: 9.3% vs. 25.9%, *p* = 0.001; junior: 9.3% vs. 52.8%, *p* < 0.001).

The article "The added value of color parameter imaging for the evaluation of focal liver lesions with “homogenous hyperenhancement and no wash out” on contrast enhanced ultrasound" was published in 2024. Journal: Front Oncol.

**Figure 4:** Diagnostic confidence score of CEUS+CPI and CEUS. CEUS, contrast-enhanced ultrasound; CPI, color parameter imaging. **(A)** displayed the diagnostic confidence scores of the senior group. There were significant differences in the number of score-1, 3, and 5 between CEUS and CEUS+CPI (4.6% vs. 28.8%, *p* < 0.001; 25.9% vs. 9.3%, *p* = 0.001; 14.8% vs. 43.5%, *p* < 0.001). **(B)** presented the diagnostic confidence scores of the junior group. There were significant differences in the number of score-1, 3, and 5 between CEUS and CEUS+CPI (1.9% vs. 22.2%, 52.8% vs. 9.3%, 2.8% vs. 28.7%, all *p* < 0.001).

### Nomogram construction

In the univariate analysis (**Table 5**), four candidate variables, namely, eccentric enhancement (senior: 70.0% vs. 29.2%, *p* < 0.001; junior: 66.7% vs. 25.0%, *p* < 0.001), feeding artery (51.7% vs. 4.2%, *p* < 0.001; 45.0% vs. 2.1%, *p* < 0.001), mosaic enhancement (63.3% vs. 6.3%, *p* < 0.001; 60.0% vs.12.5%, *p* < 0.001), and red ingredients >1/3 (90.0% vs. 14.6%, *p* < 0.001; 85.0% vs. 10.4%, *p* < 0.001) were significantly associated with M-FLLs in the senior and junior groups. Six candidate variables, namely, centripetal enhancement (senior: 43.8% vs. 18.3%, *p* = 0.004; junior: 54.2% vs.20.0%, *p* < 0.001), peripheral nodular enhancement (54.2% vs. 1.7%, *p* < 0.001; 50.0% vs. 1.7%, *p* < 0.001), subcapsular vessels (12.5% vs. 0.0%, *p* = 0.004; 10.4% vs. 0.0%, *p* = 0.015), spoke-wheel vessels (25.0% vs. 5.0%, *p* = 0.003; 18.8% vs. 6.7%, *p* = 0.021), branched vessels (22.9% vs. 5.0%, *p* = 0.006; 16.7% vs. 3.3%, *p* = 0.022), and blue and pink ingredients >2/3 (85.4% vs. 10.0%, *p* < 0.001; 89.6% vs. 15.0%, *p* < 0.001) were significantly associated with B-FLLs.

**Table 5:** Univariate analysis of identification of different features on CPI by senior and junior radiologists.

CPI feature	Senior			Junior		
	M-FLL (*n* = 60)	B-FLL (*n* = 48)	*P*-value	M-FLL (*n* = 60)	B-FLL (*n* = 48)	*P*-value
Centripetal	11 (18.3)	21 (43.8)	**0.004**	12 (20.0)	26 (54.2)	**< 0.001**
Eccentric	42 (70.0)	14 (29.2)	**< 0.001**	40 (66.7)	12 (25.0)	**< 0.001**
Centrifugal	8 (13.3)	7 (14.6)	0.852	7 (11.7)	8 (16.7)	0.455
Peripheral nodular	1 (1.7)	26 (54.2)	**< 0.001**	1 (1.7)	24 (50.0)	**< 0.001**
Feeding artery	31 (51.7)	2 (4.2)	**< 0.001**	27 (45.0)	1 (2.1)	**< 0.001**
Subcapsular vessel	0 (0)	6 (12.5)	**0.004**	0 (0)	5 (10.4)	**0.015**
Spoke-wheel vessels	3 (5.0)	12 (25.0)	**0.003**	4 (6.7)	9 (18.8)	**0.021**
Mosaic/chaotic	38 (63.3)	3 (6.3)	**< 0.001**	36 (60.0)	6 (12.5)	**< 0.001**
Branched vessels	3 (5.0)	11 (22.9)	**0.006**	2 (3.3)	8 (16.7)	**0.022**
Blue and pink ingredients >2/3	6 (10.0)	41 (85.4)	**< 0.001**	9 (15.0)	43 (89.6)	**< 0.001**
Red ingredients > 1/3	54 (90.0)	7 (14.6)	**< 0.001**	51 (85.0)	5 (10.4)	< **0.001**

CPI, color parameter imaging; M-FLL, malignant focal liver lesion; B-FLL, benign focal liver lesion. The bold values are statistically significant values that are less than 0.05.

The article "The added value of color parameter imaging for the evaluation of focal liver lesions with “homogenous hyperenhancement and no wash out” on contrast enhanced ultrasound" was published in 2024. Journal: Front Oncol.

Among them, peripheral nodular enhancement (*P* < 0.001), spoke-wheel vessels (*P* < 0.001), and red ingredients >1/3 (*P* = 0.021) were identified as independent risk factors for differentiating benign from M-FLLs by the subsequent multivariate regression analysis (**Table 6**). Thereafter, a nomogram was developed by incorporating these three predictors (**Figure 5**).

**Table 6:** Logistic regression analysis for CPI features. .

Characteristic	OR	95% CI	*P*-value
Peripheral nodular	0.01	0.00, 0.08	< 0.001
Subcapsular vessel	0.00		> 0.9
Spoke-wheel vessels	0.05	0.01, 0.25	< 0.001
Red ingredients > 1/3	6.08	1.24, 28.5	0.021

CPI, color parameter imaging; OR, odds ratio; CI, confidence interval.

**Figure 5:** Nomogram for predicting the probability of benign and malignant focal liver lesion. The range of the total points for the nomogram is 0 to 260.

### Prediction model performance assessment

The resulting model was internally validated using a 100-shot sample iterative bootstrap validation method. The degree of differentiation was assessed with the *C*-index. The model showed favorable discrimination with a *C*-index of 0.937, and the optimal diagnostic threshold value was 0.740 (0.983, 0.850) (**Figure 6A**). The calibration curve shows good agreement between the model predictions and the actual observations (**Figure 6B**).

**Figure 6:** The discrimination and calibration of the nomogram utilized for distinguishing between benign and malignant focal liver lesions. **(A)** Receiver operator characteristic (ROC) curve of the nomogram. **(B)** Calibration curve. The calibration curve effectively demonstrates the level of agreement between the predicted probabilities and the observed probabilities. The black solid line in the calibration curve represents the predictive performance of the nomogram, with a closer fit to the ideal line indicating superior prediction capabilities. AUC, the area under the ROC curve.

### Decision curve analysis

The DCA results for the nomogram are presented in **Figure 7**. In the DCA, the model offered a net benefit over the treat-all-patients scheme or the treat-none scheme at a threshold probability 5%–93%, which indicated that the application of CPI through rendering weighted features of CEUS for FLLs was very valuable for clinical practice (**Figure 7**).

The article "The added value of color parameter imaging for the evaluation of focal liver lesions with “homogenous hyperenhancement and no wash out” on contrast enhanced ultrasound" was published in 2024. Journal: Front Oncol.

**Figure 7:** Decision curve analysis depicting the clinical net benefit of the CPI nomogram.

## Discussion

FLLs can be accurately diagnosed by percutaneous needle biopsies, but studies have shown that the first biopsy was positive in 70% of patients with HCC, and puncture should be avoided in hepatic hemangioma (15, 16). When CEUS features are atypical, the diagnosis of FLLs becomes difficult, and the diagnostic confidence will be reduced. Through our research, we found that CPI could display more perfusion characteristics of lesions based on CEUS examinations. The diagnostic efficiency and diagnostic confidence could be improved. A diagnostic nomogram model based on the results of CPI features was established. This prediction model was successfully validated for the prediction of benign and M-FLLs.

CEUS provided more information about the perfusion of FLLs and improved the detection and characterization of FLLs (3, 4, 17). Many guidelines have recommended the diagnostic criterion of FLLs using CEUS in clinical practice (2, 4, 18–21). Previous studies have reported M-FLLs, especially well-differentiated HCC, and most solid B-FLLs do not wash out during the late phase (22, 23). Von Herbay et al. reported a study on the differentiation between malignant and B-FLLs in 317 patients and showed that 68% of benign and 7% of M-FLLs did not wash out during the late phase. The results showed that 93.3% of the M-FLLs were HCC (3). HCC was the only malignant lesion that might have an isoechoic appearance in the late phase, and the lack of washout caused a misdiagnosis of a benign lesion (4, 24). Another study showed that most of the M-FLLs that did not wash out in the late phases were well-moderately differentiated HCC (25). This is consistent with our study; in our study, all M-FLLs were HCC. In addition, 80.6% of the pathologically confirmed HCCs were well-moderately differentiated HCCs. The possible reason could be that the well-differentiated HCC consisted of a trabecular pattern of cell cords and rich sinusoids that may lead to stagnation and slow clearing of microbubbles. Kitao et al. suggested that the main drainage vessels in HCC switch from hepatic veins in well-differentiated tumors to hepatic sinusoids with moderate differentiation and then to portal veins (26).

The new CPI can overcome the disadvantages of CEUS and offer higher temporal resolution, more figurative images, and more objective color-coded maps in the detection of vascular morphology. The reproducibility of the CPI characteristics of our randomly selected 10 lesions was excellent and perfect (ICC: 0.830-1). The ability of CPI to diagnose FLL is consistent across radiologists and is stable and reproducible. The interobserver agreement for the CPI features was mostly excellent and perfect (k values: from 0.724 ± 0.069 to 17 0.904 ± 0.095). In our study, the AUCs of CEUS+CPI were significantly higher than those of CEUS alone (senior: 0.925 vs. 0.823, *p* = 0.037; junior: 0.818 vs. 0.653, *p* = 0.001). And CEUS+CPI by junior radiologist had comparable diagnostic performance to CEUS by senior radiologist, especially the AUC was very close (0.818 vs. 0.823, *p* = 0.520). A diagnostic prediction model of CPI for differentiating benign and M-FLLs was established. The nomogram showed good calibration and discrimination with *C*-index of 0.937. It could be used as a tool to help differentiate benign and M-FLLs with “homogenous hyperenhancement and no wash out” on CEUS. According to these results, CPI had the following advantages: (1) CPI can display the color/time distribution inside the tumor more precisely and provide more accurate information in the evaluation of lesion features. For lesions that are difficult to diagnose with CEUS, CPI substantially improved the diagnostic performance and diagnostic confidence. (2) Due to the limited clinical experience of junior doctors, the accuracy of CEUS diagnosis in junior doctors was not high. A prolonged learning process is required to achieve similar diagnostic performance with senior radiologists on CEUS (27). The addition of CPI could improve the diagnostic accuracy of junior doctors. (3) CPI analysis is a kind of postprocessing analysis technology installed in ultrasonic diagnostic equipment, so it does not increase the economic burden and examination time of patients. (4) The process of adding CPI to the practice of CEUS was very simple, but the accuracy of diagnosis was greatly improved. Several papers have evaluated the role of CPI in the diagnosis of FNH, HCC, and hepatitis infection (9, 28, 29). To date, the role of the new generation of CPI techniques with more colors and higher temporal resolution in the differential diagnosis of FLLs with the same CEUS findings—”homogenous hyperenhancement and no wash out”—has not been reported before.

The article "The added value of color parameter imaging for the evaluation of focal liver lesions with “homogenous hyperenhancement and no wash out” on contrast enhanced ultrasound" was published in 2024. Journal: Front Oncol.

According to the previous reports and our analysis, we found important features of FLLs on CEUS that are inconspicuous and ambiguous visualized by eyes can be discerned well on the images rendered by using CPI, namely, centripetal perfusion, eccentric perfusion, centrifugal perfusion, peripheral nodular enhancement, feeding artery, subcapsular vessel, spoke-wheel vessels, mosaic enhancement, branched vessels, and blue and pink ingredients >2/3 or red ingredients >1/3 (6, 7, 10, 11, 14).

The characteristics of FLLs on CPI were related to the pathological features of the lesions. Several studies have found that there is a “mosaic” in HCC (6, 7). This phenomenon occurred due to the increased tumor vascularity. The increased tumor vascularity may result from sprouting angiogenesis or recruiting existing vessels into the expanding tumor mass (30). Other studies reported that hepatic arterial supply increased and vascular abnormalities presented in HCC, such as arterialization and sinusoidal capillarization (31, 32). The feeding artery is also a feature of HCC (6, 10). Additionally, we found another specific enhancement pattern in HCC: eccentric enhancement. On the other hand, hemangiomas with arteriovenous shunts show rapid homogeneous hyperenhancement in the arterial phase. Therefore, hemangiomas can be confused with FNH, hepatic adenoma, or HCCs (4, 33). In a study by Dietrich et al., 17% (10/58) of hemangiomas had similar findings as malignant lesions (33). In our study, the better temporal resolution of CPI allowed us to visualize more peripheral nodular enhancement on CPI. The diagnosis and differential diagnosis of hepatic adenoma and HCC were analyzed in several previous studies (7, 14, 34, 35). Some studies have proposed that “pseudocapsular” or “subcapsular vessel” are commonly seen in hepatic adenomas (7, 14). In our study, “subcapsular vessel” was a specific manifestation of adenomas on CPI (senior: 6/6, 100%; junior: 5/6, 83.3%) and the “subcapsular vessel” was only present in hepatic adenomas. In FNH, spoke-wheel vessels were also easily and clearly observed on CPI images.

In this study, the DCA showed that after the application of CPI, the CEUS+CPI for the evaluation of FLLs had significantly high performance than that using CEUS alone, with risk thresholds between 5% and 93%, and this suggests that the weighted features rendered by using CPI can generate high net benefits. This further enforces the performances of AUCs obtained from ROC curves in regard to the usage of CPI.

This study had several limitations. First, our comparative analysis was conducted from retrospective research. Second, the number of lesions was small to show the benefits in some subgroup analyses, and further studies with a larger sample size are needed.

In conclusion, for FLLs with “homogeneous hyperenhancement in the arterial phase and no washout in the late phase,” CPI can better display the hemodynamic characteristics of lesions, which provides additional information for CEUS evaluation of benign and M-FLLs. Comparing to read the CEUS of the FLLs with features of “homogenous hyperenhancement and no washout” alone, a combining read of the CEUS and CPI can improve significantly the diagnostic performance of CEUS for FLLs, for the CPI can detect and render substantially subtle information of the main features of FLLs on the CEUS, and it is conducive to the radiologist for study. Future studies that expand the sample size and implement multicenter external validation are intended.

The article "The added value of color parameter imaging for the evaluation of focal liver lesions with “homogenous hyperenhancement and no wash out” on contrast enhanced ultrasound" was published in 2024. Journal: Front Oncol.

## Data availability statement

The raw data supporting the conclusions of this article will be made available by the authors, without undue reservation.

## Ethics statement

This retrospective study was approved by the Institutional Review Board of the Peking University School of Oncology (2021KT77). The studies were conducted in accordance with the local legislation and institutional requirements. The written informed consent of CEUS examination was obtained for all patients. Data collection and analysis received institutional review board approval, and the requirement for informed consent was waived.

## Author contributions

Z-NL and SW contributed equally to the paper. All authors contributed to the article and approved the submitted version.
